# Characteristics of Physical Activities and Environmental Factor Preferences of Older Adults in Rural Resettlement Community in Ningbo, China

**DOI:** 10.1155/2022/5414384

**Published:** 2022-09-10

**Authors:** Shanshan Wu, Weibo Wu, Xiuming Xia, Jingjing Zhou

**Affiliations:** ^1^School of Design, NingboTech University, Ningbo 315000, China; ^2^Qixin College, NingboTech University, Ningbo 315000, China

## Abstract

As physical mobility declines, older adults become increasingly dependent on their living environment. The relationship between physical activities and community environments for older adults has been studied to help promote physical and mental health and increase social connections among older adults, thereby improving their quality of life and health status. This study analyzed the daily outdoor physical activities of older adults in Nanyu New Village, China, using behavior mapping and questionnaire research for data collection, and conducting a comprehensive analysis of the spatial, temporal, and environmental elements of the physical activities. This research showed that the physical activity choices of older adults in rural resettlement neighborhoods vary significantly by time, gender, and space. In decreasing order, surrounding support, site security, space convenience, beautiful landscape, and diverse facilities influence the outdoor physical activities of older adults. This study provides new insights into the ongoing debate on age-friendly communities and provides a useful reference for the design of age-friendly retrofitting of outdoor environments in rural resettlement communities.

## 1. Introduction

China officially entered an aging society in 1999, and at the end of 2020, 18.7% of the total population was aged 60 and over, while 13.5% of the total population was aged 65[1]. In preparation for an aged society, the Chinese government has put forward the strategic goal of an age-friendly society and has implemented a series of national strategies [2], with age-friendly communities having become the focus [3–5]. As the physical mobility of older adults declines, mobility impairments emerge and the radius of daily physical activities gradually decreases, with older adults becoming increasingly dependent on their living environment [6, 7]. Most older adults prefer not to leave their familiar neighborhoods [8], and the outdoor spaces near their homes support them to live independently in the community and at home for as long as possible. Older adults have different expectations of their living environment than other age groups, and a good residential outdoor space provides them with access to nature [9] and a variety of opportunities for exercise, recreation, and social interaction, thereby promoting physical function [10, 11], improved mental health [12, 13], stress relief [14, 15], and longer life expectancy [16] and further fostering a sense of belonging or community [17, 18]. The recent COVID-19 health crisis has particularly affected older adults [19, 20], who have experienced the longest period of social isolation, with their range of physical activities being further reduced [21] and the neighborhood environment having a more significant impact on their daily physical activities. It is, therefore, important to understand how older adults interact with their neighborhood environment.

Since the beginning of the economic reforms in 1978, China has experienced rapid urban growth. With the rapid expansion of urban space, large amounts of rural land have been developed. As a result, former farmers have lost their farmland and have passively become urban citizens. To resettle these “new urban citizens,” the Chinese government has built a large number of rural resettlement communities (RRCs) in and around these expropriated lands, which constitute a special type of integrated urban-rural community with common characteristics of both rural and urban areas [22–26]. Compared to other urban residential areas, most older adults in RRCs have lower incomes and cannot afford to pay for a wide range of elderly care services [23]. Interaction with neighbors in outdoor spaces is an important part of these older adults' efforts to combat loneliness and enrich their daily lives [27, 28]. The small size of homes in RRCs [23] means that outdoor spaces often become an extension of older people's private living spaces and facilitate social interaction. The limited indoor living space and necessary social connections increase the demand for open neighborhood spaces for older residents in RRCs. In recent years, the Chinese government has introduced a large number of policies to promote the renovation of outdoor spaces in older neighborhoods, with RRCs being an important target for renovation [29]. Therefore, aging-friendly research for outdoor environments in RRCs is essential [30].

Previous studies have focused on older people's perceptions of the spatial environment of their community [31–33], their motivation to participate in physical activities [23–25], and the content of their physical activities [34, 35]. In more recent studies, there has been an increasing interest in the role of environmental variables [36]. The majority of such studies have focused on walking [37, 38], sightseeing [39], and physical activity [40–42], and have concentrated on developed cities in Western countries. Fewer studies have addressed the characteristics of older people's physical activities in outdoor spaces in Chinese RRCs; quantitative comparisons of the multiple environmental elements needed by older people are rare, and research on planning and design for renewal and regeneration based on the actual physical activities, characteristics, and needs of older people is not yet complete.

This study was conducted in Nanyu New Village (NNV), a rural resettlement community in Ningbo, China, to address the following questions, using the physical activity of older adults as an entry point: (1) What are the spatial and temporal characteristics of physical activity of older adults in a typical RRC in China? (2) What are the community environmental factors that influence the physical activity of older adults? (3) How community environmental factors differentially affect physical activity in older adults. The results of this study may be useful in helping designers and practitioners understand the relationship between outdoor physical activity and environmental factors so that effective interventions can be developed to promote the active use of community outdoor spaces by older adults.

## 2. Materials and Methods

### 2.1. Study Area

Ningbo is an important port city on the southeast coast of China, located in the Yangtze River Delta Economic Zone, one of the most economically developed city cluster in China, with a population of over nine million. By the end of 2020, there were 1,702,600 registered elderly people aged 60 and above in Ningbo, accounting for approximately 18.1% of the total population [43], and the degree of aging is basically on par with the national average.

Nanyu New Village (NNV) in Ningbo was used as a typical case for this study (see Figure 1), mainly for the following reasons: (1) Built-in 2005, NNV is one of the earliest demolition and rural resettlement communities in Ningbo and has a certain degree of popularity and representativeness. (2) NNV has distinctive characteristics of the rural resettlement community [44]. NNV is a gated community consisting of 31 five-story residential blocks, an activity center, and a kindergarten. The buildings in the area are laid out in rows, with a central square. The roads in the area are not smooth and surface parking is mostly used. The public green space is mainly planted with turf and shrubs, with few leisure and recreational facilities or public service facilities. (3) The proportion of elderly people in the district is high, with approximately 500 people over 60 years of age, accounting for about 25% of the total population, which exceeds the average level in Ningbo [43], and the vast majority of them are landless farmers. (4) The activity space in the district is used frequently, with a large number of people and types of physical activities, which can reflect the relationship between different types of physical activities and different spaces in a more comprehensive way.

### 2.2. Data Collection

Universal characteristics are accumulated from individual activities, so studying the physical activities of older adults from a micro-location perspective can help provide insight into the complexity and dynamics of older adults' physical activities. We used a behavior mapping approach to track older adults' physical activities and explore their active preferences. Behavior mapping is an objective tool that is widely used by researchers to study people's behavior in open spaces, such as urban streets, parks, schools, and communities, by watching different physical activities in selected locations without observer interventions to identify the association between users' behavioral patterns and implicit tendencies and certain environmental settings and spaces [45–52]. Several studies have combined behavioral mapping and GIS-supported techniques [39, 53] thus maximizing the opportunities for more sophisticated spatial analysis of the data.

The nine different physical activities of older adults that were observed were grouped into four types of physical activities (Figure 2). The first type describes physical activities related to the health of older adults. These physical activities mainly consisted of walking on the activity field, dancing in the playground, or exercising with fitness equipment. The second type of physical activity was social interaction. These physical activities mainly consisted of older adults getting together to sit or stand and chat. The third type of physical activity was life related and mainly included looking after grandchildren outdoors and doing household chores such as laundry, drying clothes, and cleaning. The fourth type of physical activity was recreational, which included doing things to relax such as sitting on a bench and contemplating or watching others, playing chess with a partner, or planting flowers.

The data for this study were collected between May and June 2021, at the turn of the spring and summer in Ningbo, when the outdoor temperature, sunshine and wind speed are suitable for outdoor physical activities for older adults.

This behavioral observation was divided into two phases. First, initial observations of the outdoor environment and the physical activities of older adults in the community were carried out in May. Based on the spatial characteristics, we divided these spaces into three categories (see Figure 3): Open, boundary, and nodal spaces. Open spaces are the central squares of the RRC, boundary spaces are adjacent to buildings, riverbanks, or road boundaries, and the spaces at the intersection of the road and residential units are defined as nodal spaces.

The formal observations took place in June. The observation period was chosen as one sunny weekday and one sunny weekend day, with 12 periods per day from 7 : 00 a.m. to 12 : 00 p.m., 2 : 00 p.m. to 6 : 00 p.m., and 6 : 00 p.m. to 9 : 00 p.m. The period of 12 : 00 p.m. to 2 : 00 p.m. was dedicated to lunch and rest time for the seniors, who rarely go outdoors, so this time was not included. Four surveyors were assigned to four areas to facilitate observations, and they stayed in each activity space for approximately 5–10 min, recording all older adults present and moving around. Each observer used a timer and mobile phone camera to collect data, specifically the number, gender, and time of various physical activities, which were recorded on prepared recording sheets and maps, and then the original hand-drawn observations were digitally recorded in a GIS mapping system using SuperMap iDesktop 8C.

Ten older adults were also randomly selected for interviews during the initial observation phase to determine which elements they needed. Based on the NNV survey and interviews, together with the analysis of various design guidelines [54–57] and published studies [14, 33, 58–66], 15 environmental elements (Table 1) were finally selected to design a questionnaire. The first part of the questionnaire included basic information about the participants and their most common choice of outdoor physical activities. The second part of the questionnaire rated the importance of older people on 15 environmental factors that influence their participation in outdoor physical activities (from 1 = not at all important to 5 = very important).

Then, during the formal survey, the observers randomly distributed 5–10 questionnaires in each activity space in NNV, each completed under the supervision of the observers. A total of 100 questionnaires were distributed and 83 valid questionnaires were returned, resulting in a completion rate of 83%.

### 2.3. Data Analysis

SPSS Statistics V22 was used to create a database of outdoor physical activities of older adults in NNV. Descriptive statistics and chi-square tests were used to compare the activity categories and differential characteristics by gender, activity time, and activity date. The activity data from the two-day observations were entered into the GIS platform and the spatial characteristics of the residents' outdoor physical activities were identified through GIS's kernel density analysis.

The volume of physical activities participated in does not provide a complete picture of the level of participation in physical activities. Therefore, this study used the volume of physical activities, the duration of physical activities, and the fluctuations of physical activities to obtain the participation index (Pi) for each activity, to provide a comprehensive picture of the level of participation of older adults in physical activities.

The volume of activity (Va) is the average number of participants in each type of activity on the day of observation and reflects the number of physical activities participated in.

The duration of physical activities (Da) is defined as the ratio of the number of periods in which the activity occurs to the total number of statistical periods as the duration value, reflecting the degree of continuity of activity participation. [65].

(1) $$\begin{array}{c} D_{a}=\frac{D_{n}}{D_{s}}. \end{array}$$

Fluctuations of activity (Fa) indicate the stability of activity participation [65]; the less volatile the data, the more stable they are. Fa is judged by analyzing the difference between the maximum and minimum values of activity as a percentage of the mean.

(2) $$\begin{array}{c} F_{a}=\frac{\left(V_{max}-V_{min}\right)}{V_{avg}}. \end{array}$$

To make the values of the different measures comparable, the number of physical activities, the duration of the physical activities, and the stability of the physical activities were normalized using a linear function normalization method (3), i.e., the raw data were converted into a range of values [0,1] by isometric scaling:

(3) $$\begin{array}{c} Y_{\text{norm}}=\frac{Y-Y_{\text{min}}}{Y_{\text{max}}-Y_{\text{min}}}. \end{array}$$

Expert scoring and statistical averaging were then used to determine the weight values of the indicators [47, 66]. Ten experts in the field of study were invited to rate the indicators in this study. Each expert was given 100 points and assigned to each indicator based on his judgment of the importance of participation in outdoor physical activities. The weight values for each indicator were then calculated and standardized based on the average score of the 10 experts (see Table 2). The participation index of the physical activities was quantified by a weighted average of these three indicators.

(4) $$\begin{array}{c} \text{Pi}=0.65\times \text{Va}+0.23\times \text{Da}+0.12\times Fa. \end{array}$$

Factor and correlation analyses were conducted on the questionnaire data using SPSS. The degree of importance of the relevant environmental elements was compared by the level of participation in outdoor physical activities of older adults, i.e., the higher of participation index in the activity, the more important the elements associated with the activity [67].

## 3. Results

### 3.1. Outdoor Physical Activities for Older Adults

A total of 1524 physical activities were recorded over two days on weekday and weekend in NNV. Among the types of outdoor physical activities for older adults (see Figure 4), social physical activities were selected by the highest percentage at 54.5%, followed by recreational physical activities at 31.6%. Life-related physical activities and health-related physical activities were less frequently selected at 7.1% and 7.0%, respectively.

Descriptive statistics and chi-square tests revealed that there was a significant difference in the choice of outdoor physical activities by gender (*p*  = 0.000 < 0.01) (see Table 3). The overall number of female seniors who were active outdoors was higher than that of male seniors. A comparison of the differences in the percentages showed that 60.60% of females chose social interactive physical activities, which is significantly higher than the 44.75% of males. The percentage of men choosing recreational physical activities was 47.80%, significantly higher than the percentage of women choosing them (21.31%). The weekday and weekend showed a nonsignificant difference (*p*  = 0.164 > 0.05) for the type of activity. Most of the elderly people in the rural resettlement community were landless farmers and were mostly unaffected by their weekday. However, the number of elderly people who were active on a weekday was higher than that on weekend.

The chronological curve of outdoor activity for older adults as a whole (see Figure 5) show three peaks—at 9 : 00 a.m., 3 : 00 p.m., and 7 : 00 p.m., respectively—with a trough at 11 : 00 a.m.

The chronological variation in health-related physical activities differed significantly from the others (see Figure 6), with the peak occurring at 7 : 00 p.m., dominated by square dancing, with some other fitness activity before 9 : 00 a.m. and a persistent low in the afternoon. Social interactive activity was the dominant outdoor activity, mainly chatting, and it showed the same characteristics as the overall chronological curve change. The temporal variation in life-related physical activities differed significantly between weekdays and weekends, with the same peak in the morning on weekdays and weekends, mainly for chores such as childcare and washing and drying. There was also another peak at 3 : 00 p.m. on the weekend, mainly for childcare, with fewer household physical activities and overall lower activity than the morning peak, while the other peak on weekdays was lower at 6 : 00 pm, mainly for household physical activities such as cooking and tidying. Recreational physical activities had a more moderate morning and afternoon peak during the day, with a higher concentration of activity between 8 : 00 a.m. and 9 : 00 a.m. and between 2 : 00 p.m. and 3 : 00 p.m., with watching being the main activity, more evenly spread throughout the day, and chess being significantly more concentrated in the afternoon.

Physical activities, such as chatting, childcare, and housework, were significantly more common among females than male seniors (see Figure 7), with female seniors preferring to spend their mornings and evenings engaging in health-related physical activities and life-related physical activities, such as dancing, gym equipment, and housework, while male seniors preferred to spend their mornings and afternoons with pastimes such as chess, watching, and gardening.

The chi-square test (see Table 4) revealed significant differences in the outdoor physical activities of older adults in the different spatial types (*p* = 0.000 < 0.01). The kernel density from GIS showed a clear clustering of older adult physical activities and an uneven distribution of activity types (see Figure 8). There is one open space in the NNV, the central square, where the density of people was high and the frequency of the four types of activity was relatively even. The boundary spaces were less densely populated, with recreational physical activities accounting for 59.2%. The boundary space near the activity center building forms an obvious density center, followed by the residential boundary in the southwest corner and the boundary along the river in the northwest corner, where crowd activities are more dispersed. The nodal space was the most dominant activity space for older adults, accounting for 65.4% of the total number of physical activities. Social interactive physical activities (64.7%) were the main types of activity in this location. Lifestyle physical activities (4.7%), although of a relatively small proportion, occurred more frequently than in other spaces. Multiple obvious density centers appear in the nodal space, mainly concentrated in the south-central area of the neighborhood.

### 3.2. Analysis of Factors Affecting Outdoor Physical Activities of Older Adults

This study collected 83 valid questionnaires: 48 (57.8%) were female and 35 (42.2%) were male. A total of 6% of the older adults lived alone, 32.5% lived with their spouse, and the rest lived with their children. Meanwhile, 96.4% of the older people who participated in this survey had lived in NNV for more than one year, and 78.3% had lived there for more than five years. Older people who took part in this survey were active outdoors, with 45.8% participating more than once a day, 31.4% participating three to four times a week, and 22.9% participating once a week or less.

In the exploratory factor analysis, the results of the KMO and Bartlett's tests showed a sufficient value of 0.808 (0.5< KMO <1) and a significance of 0.000 < 0.05, which indicates qualified data for the next analysis (see Table 5). The rotated component matrix was divided into five groups based on its loading on each factor (see Table 6).

Factor 1 was named space convenience because it includes number of spaces, generous areas, spatial diversity, and spatial accessibility, which, together, determine the characteristics of space and reflect the needs of older adults for activity spaces. Factor 2, which includes tables and chairs, shelter from sunshine/rain, and lighting, reflects the need for environmental support for older adults and was, therefore, named surrounding support. Factor 3 was named site safety, as it includes elements such as barrier-free facilities, hygiene environment, secure ground, and pedestrian paths, reflecting the need for site safety for older adults. Factor 4 includes vegetation and landscape pieces, reflecting the need for landscaping for older adults, and was therefore named beautiful landscape. Factor 5 includes fitness facilities and children's facilities, reflecting the need for activity facilities for older adults, and was, therefore, named facility enhancement.

### 3.3. The Importance of Environmental Elements Based on the Needs of the Elderly

A correlation analysis was conducted between the importance of environmental elements and outdoor physical activities for seniors (see Table 7). There was a wide variation in the correlations between older adults' physical activities and the 15 environmental factors. Number of spaces, children's facilities, and landscape pieces were not correlated with any of the physical activities for older adults. Lighting was correlated with four physical activities: chatting, dancing, cards and chess, and gardening. Most of the other elements were significantly correlated with one to two physical activities.

Health-related physical activities were positively influenced by spatial diversity, fitness facilities, lighting, secure ground, barrier-free facilities, and vegetation (see Figure 9). Social interactive physical activities were significantly correlated with spatial accessibility and lighting. Life-related physical activities were positively influenced by the generous area, tables and chairs, vegetation, and hygiene environment. Recreational physical activities were influenced by tables and chairs, shelter from sunshine/rain, barrier-free facilities, secure ground, pedestrian paths, and lighting.

The importance of the relevant environmental elements was determined by the level of the participation index of each activity, with a higher activity participation index indicating a greater importance of the relevant element. The participation indexes of the physical activities after normalization are shown in Table 8. The highest Pi was chatting (0.997), followed by watching (0.675), childcare (0.357), walking (0.240), housework (0.216), cards and chess (0.182), using fitness equipment (0.091), gardening (0.090), and dancing(0.036).

As can be seen in Table 9, the impact scores of each element and each factor toward the physical activities of older adults were disclosed.  Figure 10 illustrates the importance of the various influencing elements. Environmental support takes the most important role with the highest score (3.012), descending in order as follows: site safety (2.636), space convenience (1.508), beautiful landscape (0.597), and diverse facilities (0.091).

## 4. Discussion

### 4.1. Characteristics of the Outdoor Physical Activities for Older Adults

The peak physical activity periods for older adults are concentrated at 9 : 00 a.m., 3 : 00 p.m., and 7 : 00 p.m., which is largely consistent with other studies [44, 68]. The peak in health-related physical activities occurred at 7 : 00 pm and was dominated by square dancing. Social interactive activity was the dominant outdoor activity, which showed the same peak as overall. Life-related physical activities peaked at 9 : 00 a.m., while recreational physical activities experienced a more moderate peak during the day.

This study found nonsignificant differences in the types of physical activities older adults engage in on weekdays and at weekends. Still, there were a few differences in some physical activities. For example, housework was significantly higher at 6 : 00 p.m. on the weekend than on a weekday, and the amount of childcare were higher on a weekday than on weekend. An analysis of the comments received during the survey showed that the amount of weekday childcare is higher mainly because older adults in China need to help their children with childcare during the week. Most children come to NNV to visit the elderly on the weekend and have dinner together in the evening, so the number of household physical activities spent by the elderly on preparing dinner was also elevated.

In terms of gender, older female adults tend to be more active in social interactive and life-related physical activities such as chatting, childcare, dancing, and housework, while older male adults prefer to engage in recreational physical activities, such as playing cards and chess, watching, and gardening, similar to the findings of some previous studies [40, 44, 69]. Overall, females tend to be more active within NNV than males. The possible reasons for this are that older Chinese men have a greater range of daily physical activities than women and use urban public facilities and spaces more than older women [68], while older women are more dependent on community spaces [69]. In addition, square dance physical activities are more popular among older Chinese women than men.

Open space in NNV is the central square, where seniors have the most diverse types of activities. This space is large, flat, and open, with fitness equipment, where the elderly enjoy dancing and exercising, and where 90% of the health-related physical activities in NNV take place. There are several seats and lounge kiosks, where chatting and watching take place more frequently, and there are a certain number of grandchildren using the children's facilities.

Boundary spaces that are close to public buildings with high pedestrian traffic or street spaces are more attractive to older adults, while spaces between houses close to residential buildings are often occupied by vehicles and appear constricted and passive, with fewer physical activities for older adults. Boundary spaces have strong boundaries and tend to encourage resting and playing cards and chess. The density of people moving around here is low, and recreational physical activities such as cards and chess are mainly played in groups of two to five people, which attracts other people to gather around. The presence of pedestrians and active people in the boundary space increases the sense of participation of the elderly.

Due to the deterioration of the physical mechanisms of the elderly, the scope of their daily physical activities is concentrated in nodal spaces such as the entrances to residential units. Social and recreational physical activities are the main types of activity in this area. The high accessibility of this type of space makes it easy to attract older adults and make them congregate. However, the spaces are small in scale and the physical activities are relatively homogeneous, with small-scale conversations between one and three people. There are also some spaces where more varied physical activities occur, such as childcare, chess, and cards, creating a rich and interactive atmosphere with close communication.

### 4.2. Environmental Elements Affecting the Physical Activities of Older Adults

The environmental elements of residential areas play an important intervening role in supporting or limiting older adults' need for autonomy and independence, and a good environment can enhance their sense of access and self-confidence and positively influence health, thereby indirectly reducing pressure on public health services [66, 70].

Environmental support has the greatest impact on outdoor physical activities for older adults, whose physiological characteristics lead to a greater reliance on such elements. Older adults are susceptible to falling on wet ground. Spaces that provide shelter from the rain allow older adults to enjoy outdoor physical activities without having to worry about sudden changes in the weather. Due to their limited physical strength and health conditions, older adults are unable to engage in long periods of uninterrupted exercise or walking and are easily fatigued. Sufficient seating is needed for older adults to rest, which makes it easier for them to observe the physical activities around them and also increases the opportunity for them to talk and chat with one another—an important factor for older adults to move around in open spaces in the community [71]. Tables and chairs, shelter from sunshine/rain, and lighting provide a more comfortable place for older adults to sit and chat, play chess and cards, and engage in other specialized and companionable communication and interaction [72]. These are highly consistent with the findings of this study.

Site safety has a greater impact on aging outdoor physical activities, with older adults showing an increased emphasis on safety with age and declining physical function [73, 74]. Secure ground and barrier-free facilities are priority elements for older adults engaged in dancing and watching. Wider walking paths make it easier for older adults to pass without disturbing other pedestrians. The importance of good hygiene may be rooted in older adults' awareness that a dirty environment increases their risk of illness, and that good sanitation not only makes the environment more pleasing to the eye but also makes outdoor physical activities more enjoyable for older adults accompanying children [70, 75].

Space convenience has an impact on the quality of outdoor physical activities in old age. Proximity to home is the primary spatial consideration for older adults when engaging in outdoor physical activities, and the spatial location remains relatively important, especially for older adults with poor health and limited mobility [69]. Generous area indicates a tendency for older adults to be aggregation-oriented, with older adults preferring spacious spaces that can support a certain level of gathering. The enrichment of large and small spaces with transitions and interspersed spaces can meet the different needs of older adults under different conditions [74], allowing them the freedom to choose and diversify their living behavior patterns.

Beautiful landscapes impacted the quality of outdoor physical activities for older adults in general. The quality of vegetation in the landscape attracts older adults to outdoor physical activities and enhances the pleasure of interaction, but is not a key factor, which is not entirely consistent with other studies [70, 76, 77]. It is possible that the early year of construction of NNV, the small variety of vegetation, its rudimentary form, and the lack of maintenance have led to a lack of significant appeal for older adults' physical activities. Older adults also do not devote their attention to sculptures in the environment, and instead may feel that such amenities crowd the activity space [76].

The improvement of diverse facilities had the least impact on the outdoor physical activities of the elderly in the rural resettlement community. Although some studies have shown that fitness facilities can increase the amount of activity of older adults [59], the enhancement of children's facilities can provide a place for the old and the young to play together, increasing the intensity and pleasure of communication between the elderly and children and between the elderly [55, 77]. However, only a small number of elderly people use fitness facilities in NNV, possibly due to reasons such as the aging of said fitness facilities or their inappropriateness in terms of the physical characteristics and scale of the elderly, which can easily lead to exercise injuries, and children using play facilities may rush the elderly and cause injuries to the latter, thus making such facilities unattractive to the elderly [60].

### 4.3. Recommendations for the Optimization of Age-Friendly Environments

Based on these findings, we put forward several design recommendations: (1) Environmental support, such as lighting, seating, and shelter from sunshine/rain, are the most basic needs to support outdoor physical activities for older adults and need to be adequately safeguarded. (2) The safety of activity areas should be carefully considered, with particular attention given to their barrier-free design, and walking paths should be more personalized to suit the needs of older people, as well as avoid any corners that could lead to hygiene problems. (3) Spatial accessibility needs to be given high priority, combining spatial boundaries with natural elements, which can enrich the interest in outdoor spaces and enhance well-being. (4) The choice of fitness and children's facilities needs to be carefully decided or adapted to the environment; otherwise, they will not only take up space but also pose a safety hazard.

### 4.4. Strengths and Limitations

Field observations are more suitable than big data analysis for understanding the needs and uses of the outdoor environment of older adults at a microspatial scale. Compared to other studies, this study provided a quantitative approach to the study of outdoor spaces by exploring the importance of environmental elements more precisely based on differences in the outdoor activity characteristics and needs of older adults. However, this study has the following limitations. First, the study only included one community as the study site, so the results may be limited by the scope of the study and there is a potential risk of generalizing the results to other communities. Second, the specific locations of the observations and observation activities were recorded by hand, which may have affected the accuracy of the results even for a trained observer. Future studies may extend the scope of the study to other scales of space and environment and may even extend to different age groups.

## 5. Conclusions

With the booming urbanization in China, there is an increasing demand for outdoor spaces. The Chinese government has launched many policies to promote the transformation of outdoor community spaces, with rural resettlement communities being an important target for transformation. Older people are the main users of outdoor spaces in such communities and are also a vulnerable group in life. Therefore, research on the physical activities of elderly people in rural resettlement communities is of great relevance. This study investigated the patterns and spatio-temporal characteristics of four major categories and nine subcategories of outdoor physical activities of older people and derived the importance of environmental elements in influencing the physical activities of older people based on the participation index of outdoor physical activities. This study provided new insights into the ongoing debate on age-friendly outdoor development in China and provides a basis for the government and policymakers in planning more appropriate spaces for rural resettlement communities and promoting the construction and adaptation of activity sites. [78–83].

## Figures and Tables

**Figure 1:** Location of Nanyu new village.

**Figure 2:** Classification of physical activities for older adults in the NNV's outdoor spaces.

**Figure 3:** Three categories of outdoor spaces in NNV: (a) Open spaces; (b) boundary spaces; (c) nodal spaces.

**Figure 4:** Proportion of physical activities that occurred in the NNV's outdoor spaces.

**Figure 5:** Total elderly people using public spaces in NNV per hour.

**Figure 6:** Total number of elderly persons per hour across the four types of physical activities.

**Figure 7:** Gender differences in physical activities.

**Figure 8:** Spatial distribution of physical activities for older people in NNV. (a) Density analysis of the positions. (b) The categories and distribution of positions.

**Figure 9:** Correlation between the environmental elements and physical activities of older people.

**Figure 10:** Impact score between the environmental elements.

**Table 1:** Age-friendly physical environments in public open spaces.

1 number of activity spaces	6 secure ground	11 pedestrian path
2 generous area	7 tables and chairs	12 fitness facilities
3 spatial diversity	8 shelter from sunshine/rain	13 children's facilities
4 spatial accessibility	9 lighting	14 vegetation
5 hygienic environment	10 barrier-free facilities	15 landscape pieces

**Table 2:** Weighted values of three indicators for a combined ratio of physical activities.

Indicators	Va	Da	Fa
Weighted values	0.65	0.23	0.12

**Table 3:** Weighted values of three indicators for a combined ratio of physical activities.

Name		Activity type *N* (%)				Total	Sig. (*p*)
		Health-related physical activities	Social interactive physical activities	Life-related physical activities	Recreational physical activities		
Gender	Male	17(16.19%)	260(31.48%)	27(25.00%)	286(58.97%)	590(38.71%)	0.000^*∗∗*^
	Female	88(83.81%)	566(68.52%)	81(75.00%)	199(41.03%)	934(61.29%)	
Date	Weekday	58(55.24%)	420(50.85%)	67(62.04%)	259(53.40%)	804(52.76%)	0.164
	Weekend	47(44.76%)	406(49.15%)	41(37.96%)	226(46.60%)	720(47.24%)	

^*∗*^ *p* < 0.05; ^*∗∗*^*p* < 0.01.

**Table 4:** Chi-square test for activity type and type of space.

Type of space	Activity type N (%)				Total	Sig. (*p*)
	Health-related physical activities	Social interactive physical activities	Life-related physical activities	Recreational physical activities		
Open spaces	94 (29.2%)	125 (38.8%)	40 (12.4%)	63 (19.6%)	322 (21.1%)	0.000^*∗∗*^
Boundary spaces	6 (2.9%)	57 (27.7%)	21 (10.2%)	122 (59.2%)	172 (13.5%)	
Nodal spaces	5 (0.5%)	644 (64.7%)	47 (4.7%)	300 (30.1%)	1030 (65.4%)	

^*∗*^ *p* < 0.05^*∗∗*^*p* < 0.01.

**Table 5:** Chi-square test for activity type and type of space.

Kaiser–Meyer–Olkin measure of sampling adequacy		0.808
Bartlett's test of sphericity	Approx. Chi-square	624.317
	Df	105
	Sig.	0.000

**Table 6:** Chi-square test for activity type and type of space.

Environmental factors	Environmental elements	Component				
		1	2	3	4	5
Space convenience	Spatial diversity	**0.815**	0.277	0.172	0.126	0.150
	Generous area	**0.814**	0.097	0.209	0.264	0.116
	Number of activity spaces	**0.790**	0.209	−0.006	0.044	0.406
	Spatial accessibility	**0.707**	0.243	0.356	0.103	−0.032
Surrounding support	Shelter from sunshine/rain	0.144	**0.821**	0.095	0.272	−0.080
	Tables and chairs	0.310	**0.793**	0.116	−0.062	−0.025
	Lighting	0.234	**0.708**	0.250	−0.067	0.199
Site safety	Pedestrian paths	0.287	0.260	**0.701**	0.175	0.222
	Barrier-free facilities	−0.069	0.553	**0.631**	−0.096	0.134
	Hygiene environment	0.383	−0.046	**0.610**	0.355	0.082
	Secure ground	0.391	0.392	**0.537**	0.010	0.139
Beautiful landscape	Vegetation	0.144	0.237	0.146	**0.831**	0.139
	Landscape pieces	0.157	−0.161	0.052	**0.789**	0.280
Diverse facilities	Fitness facilities	0.130	−0.003	0.222	0.125	**0.851**
	Children's facilities	0.212	0.078	0.074	0.340	**0.759**

**Table 7:** The physical activities' correlations with environmental elements.

Environmental elements	Health-related physical activities			Social interactive physical activities		Life-related physical activities	Recreational physical activities		
	Walking	Using fitness equipment	Dancing	Chatting	Childcare	Housework	Watching	Cards and chess	Gardening
Spatial accessibility	−0.068	0.186	0.018	**0.269 ** ^*∗*^	0.194	0.087	0.205	0.087	0.186
Generous area	−0.007	0.199	0.167	0.165	**0.268 ** ^*∗*^	0.042	0.007	0.001	0.173
Number of activity spaces	0.003	0.134	0.149	0.157	0.177	0.017	0.022	0.098	0.192
Spatial diversity	0.144	**0.243 ** ^*∗*^	0.153	0.071	0.200	0.014	0.112	0.157	0.135
Shelter from sunshine/rain	0.157	0.068	0.162	0.107	0.040	0.065	**0.244 ** ^*∗*^	0.015	0.080
Tables and chairs	0.112	0.105	0.208	0.207	**0.220 ** ^*∗*^	0.068	**0.297 ** ^*∗∗*^	0.058	−0.017
Lighting	0.006	0.042	**0.231 ** ^*∗*^	**0.224 ** ^*∗*^	0.091	0.048	0.205	**0.240 ** ^*∗*^	0.245^*∗*^
Barrier-free facilities	−0.023	0.040	**0.308 ** ^*∗∗*^	0.008	0.063	−0.140	**0.276 ** ^*∗*^	0.109	0.045
Hygiene environment	0.073	0.072	−0.002	0.057	**0.228 ** ^*∗*^	−0.142	0.157	0.075	**0.233 ** ^*∗*^
Secure ground	0.079	0.131	**0.223 ** ^*∗*^	0.145	0.173	−0.102	**0.260 ** ^*∗*^	0.131	0.016
Pedestrian paths	0.115	0.106	0.114	0.155	0.168	−0.174	**0.296 ** ^*∗∗*^	**0.222 ** ^*∗*^	0.168
Fitness facilities	0.025	**0.226 ** ^*∗*^	−0.045	−0.033	0.126	−0.204	−0.154	0.204	0.066
Children's facilities	0.060	0.086	0.077	−0.042	0.092	−0.017	−0.071	0.082	0.139
Vegetation	**0.243 ** ^*∗*^	0.114	0.033	0.035	**0.267 ** ^*∗*^	−0.115	−0.032	0.177	−0.071
Landscape pieces	0.047	0.038	−0.133	−0.054	0.143	−0.060	−0.196	−0.002	−0.121

^*∗*^ correlation is significant at the 0.05 level. ^*∗∗*^ correlation is significant at the 0.01 level.

**Table 8:** The participation index of physical activities.

Type	Physical activities	Va	Da	Fa	*P*i	Ranking
Health-related physical activities	Using fitness equipment	0.220	0.333	0	0.091	7
	Dancing	0.050	0	0.032	0.036	9
	Walking	0.023	0.524	0.868	0.240	4
	Total				0.367	
Social interactive physical activities	Chatting	1	1	0.975	0.997	1
	Total				0.997	
Life-related physical activities	Housework	0.043	0.429	0.745	0.216	5
	Childcare	0.067	0.857	0.964	0.357	3
	Total				0.573	
Recreational physical activities	Watching	0.501	1	1	0.675	2
	Cards and chess	0.060	0.286	0.642	0.182	6
	Gardening	0	0.143	0.477	0.090	8
	Total				0.947	

**Table 9:** The impact of environmental elements.

Factors	Elements	Physical activities	Participation index	Impact score
Space convenience	Number of spaces	None	0	0
	Generous area	Childcare	0.357	0.357
	Spatial diversity	Using fitness equipment	0.091	0.091
	Spatial accessibility	Chatting	0.997	0.997
	Total			1.445
Environmental support	Tables and chairs	Watching	0.675	0.675
	Shelter from sunshine/rain	Childcare	0.357	1.032
		Watching	0.675	
	Lighting	Dancing	0.036	1.305
		Chatting	0.997	
		Cards and chess	0.182	
		Gardening	0.090	
	Total			3.012
Site safety	Barrier-free facilities	Dancing	0.036	0.711
		Watching	0.675	
	Hygiene environment	Childcare	0.357	0.357
	Secure ground	Watching	0.675	0.711
		Dancing	0.036	
	Pedestrian path	Watching	0.675	0.857
		Cards and chess	0.182	
	Total			2.636
Diverse facilities	Fitness facilities	Using fitness equipment	0.091	0.091
	Children's facilities	None	0	0
	Total			0.091
Beautiful landscape	Vegetation	Childcare	0.357	0.597
		Walking	0.240	
	Landscape pieces	None	0	0
	Total			0.597

## Data Availability

The data used to support the findings of this study are available from the corresponding author upon request.
